# Study on the Mechanism of circRNA-0024103 Reducing Endothelial Cell Injury by Regulating miR-363/MMP-10

**DOI:** 10.1155/2022/1709325

**Published:** 2022-08-02

**Authors:** Yunfei Tian, Guofu Zheng, Hailiang Xie, Yi Guo, Hui Zeng, Youlin Fu, Xiaochun Liu

**Affiliations:** ^1^Department of Minimally Invasive Intervention, The Affiliated Ganzhou Hospital of Nanchang University, Ganzhou 341000, Jiangxi, China; ^2^Department of Vascular and Hernial Surgery, The Affiliated Ganzhou Hospital of Nanchang University, Ganzhou 341000, Jiangxi, China

## Abstract

Cardiovascular diseases could damage the heart and blood vessels, which cause mortality and morbidity. It is of great significance to explore targeted therapeutic approaches for atherosclerosis that is one of the most common vascular lesions and the main pathological basis of cardiovascular disease. However, the function of circRNA-0024103 in cardiovascular diseases is still not clear. Therefore, we aim to observe the effect of circRNA-0024103 modulation of miR-363/MMP-10 axis on biological behaviors such as proliferation and migration of endothelial cells after ox-LDL induction. The effects on the proliferation ability of endothelial cells were observed by CCK-8 assay and EdU assay based on overexpression of circRNA-0024103 in combination with miR-363 mimic or MMP-10 siRNA, and then, the effects on apoptosis were detected by flow cytometry analysis. The effects on cell migration, invasion, and angiogenesis were further examined by scratch assay, transwell assay, and tube formation assay. The results in CCK-8 and EdU assays showed that miR-363 mimic or MMP-10siRNA significantly attenuated the proliferation-promoting effect of overexpressed circRNA-0024103 on cell proliferation. In flow cytometry assays to detect apoptosis, overexpression of circRNA-0024103 inhibited apoptosis of endothelial cells, and the intervention of combined miR-363 mimic or MMP-10 siRNA counteracted the inhibitory effect of overexpression of circRNA-0024103 on apoptosis, resulting in a significant increase in the number of endothelial cells undergoing apoptosis. The migration, invasion, and tube-forming ability of endothelial cells were significantly enhanced when circRNA-0024103 was overexpressed, while the promotion of migration, invasion, and the tube-forming ability by overexpression of circRNA-0024103 alone was counteracted when combined with miR-363 mimic or MMP-10 siRNA. circRNA-0024103 regulates the biological behaviors of endothelial cells such as proliferation, apoptosis, migration, and invasion through the miR-363/MMP-10 axis. Our finding provides a new therapeutic target for the treatment of atherosclerosis.

## 1. Introduction

With economic and social development, cardiovascular diseases have imposed a huge health and economic burden on human beings worldwide, with high mortality and morbidity rates [1]. Atherosclerosis (AS) is one of the most common vascular lesions and the main pathological basis of cardiovascular disease, characterized by the formation of complex atherosclerotic plaques, leading to atherosclerosis and stenosis, which clinically manifests as coronary heart disease, peripheral arterial disease, and ischemic stroke [2, 3]. Atherosclerosis, a chronic inflammatory disease of the arterial wall, is the primary cause of various serious cardiovascular diseases, and among the multiple mechanisms leading to atherosclerosis, endothelial damage is considered to be the primary cause. Elevated LDL is an important risk factor [4–6], and oxidatively modified LDL is more potent in promoting atherosclerosis [7]. Stenosis or vascular occlusion caused by rupture of unstable atherosclerotic plaques, platelet aggregation, and thrombosis can lead to severe cardiovascular disease, posing a great threat to human health. Therefore, it is particularly urgent to explore targeted therapeutic approaches for atherosclerosis.

In the pathogenesis of atherosclerosis, many cells and molecules are involved in its pathology and pathophysiology, including mainly endothelial cells, smooth muscle cells, and inflammatory cells[8, 9]. There are three main theories on the pathogenesis of atherosclerosis, namely the lipid infiltration theory, the endothelial injury theory, and the vascular smooth muscle cell migration and proliferation theory. Among them, the endothelial damage theory suggests that atherosclerotic plaques are the product of endothelial damage in arteries and that the pathophysiology of AS originates from endothelial cell damage, and subsequently more and more studies point to endothelial cell dysfunction as a marker of early atherosclerosis. Thus, improving the function of endothelial cells is of great importance for the treatment of atherosclerosis. Circular RNAs (circRNAs) are a new class of endogenous non-coding RNAs (ncRNAs) that do not have 5' caps and 3′ poly(A) tails and exist in their characteristic covalent closed-loop form. A growing number of studies have shown that circRNAs are widely present In Vivo, stably expressed in plasma, serum, and tissues, and involved in the regulation of eukaryotic gene expression [10, 11]. circRNA-0024103 is a newly identified circRNA that has been studied to regulate MMP-10 expression in human cartilage degradation by acting as a miR-363 “sponge,” but its function in cardiovascular disease is not yet clear. However, its function in cardiovascular diseases is not yet known.

In a study, the expression profile of cyclic RNAs in human umbilical vein endothelial cells after oxidative LDL induction was analyzed, and 943 differential cyclic RNAs with 2-fold change in expression were screened, and in functional experiments, cyclic RNAhSA_circ_0003575 silencing was found to promote the proliferation and angiogenic capacity of human umbilical vein endothelial cells and combined with bioinformatics methods to predict this cyclic RNA. This combined with bioinformatics methods predicted the miRNA targets regulated by this circRNA, revealing the existence of a regulatory network. circRNA-miRNA-mRNA in the regulation of endothelial cell function. In another study, the expression profile of cyclic RNA in endothelial cells after hypoxia treatment was examined, and among the cyclic RNAs screened, silencing the expression of the cyclic RNSAcZNF292 resulted in a significant reduction in the number of tube-forming endothelial cells cultured in vitro, thus suggesting that cZNF292 has proangiogenic activity in vitro [12].

Therefore, in this study, we investigated the role of circRNA-0024103 in the regulation of endothelial cell function and further investigated the specific mechanism of its regulatory role. We conducted an ox-LDL intervention in HUVECs cells. We also used SPSS 23.0 for data processing and analysis. The *t*-test was used for comparison between two groups of samples.

## 2. Materials and Methods

### 2.1. Ox-LDL Intervention in HUVECs Cells

The ox-LDL was prepared at different concentrations (0, 40, 60, 80, and 100 mg/l), and the optimal intervention concentration was selected by detecting the expression of circRNA-0024103 by PCR. The selected intervention concentration was then treated with HUVECs cells for different times (6 h, 12 h, 24 h, and 48 h), and again, the optimal intervention concentration was selected by detecting the expression of circRNA-0024103 expression to screen out the optimal intervention time.

The total RNA of each group of cells was extracted, reverse transcribed, and subjected to qRT-PCR. As given in Table 1, the primer sequences required for the experiments were synthesized by Shanghai Biotech Biological Co., Ltd.

### 2.2. Cell Culture and Transfection

HUVECs and HEK293 T cells were cultured in DMEM containing 10% FBS, and the cells were incubated at 37°C in a cell culture chamber with 5% CO_2_, and the culture medium was changed every 2 days. Lipofectamine 3000 was used for transfection experiments. First, cells in good growth condition were digested with trypsin and resuspended and inoculated into new well plates. The cells were removed from the incubator overnight and observed when they reached 80% confluence for the next step. Referring to the recommended measurements in the instructions, Lipofectamine 3000 and plasmid DNA are added to serum-free DMEM medium, gently mixed, and left for 20 min, and then, the mixed solution is added to the well plate for intervention. circ-0024103 overexpression plasmid pcDNA3.1 was provided by Hanheng Biotechnology Co., Ltd.

HUVECs cells were transfected with circ-0024103 overexpression plasmid as described above, and then, the cells were digested and prepared into cell suspensions. The cells were inoculated into 96-well plates with 4×10 cells per well^3^, and 6 replicate wells were set up for each group. 20 ul of CCK-8 reaction solution was added to each well at 0 h, 24 h, 48 h, and 72 h, respectively, and the cells were incubated in the incubator for 2 h, and the OD value was measured at 450 nm with an enzyme standard. HUVECs transfected with circ-0024103 overexpression plasmid were inoculated in 24-well plates overnight; EdU was prepared in the medium at a concentration of 50 mm, and 300 ul was added to each well (the amount should not be excessive, but should just cover the cells) and incubated in the cell incubator for 3 h. Afterward, the medium was discarded, and the cells were washed with PBS solution for 5 min each time. The cells were then washed with PBS solution for 5 min each time and repeated three times to elute the residual unadulterated DNA EdU, fixed, Apollo staining, DNA staining, and image acquisition.

### 2.3. Flow Cytometric Detection of Apoptosis

Prepare 10× binding buffer with deionized water to a final concentration of 1× binding buffer solution; digest the cells gently with 0.25% EDTA-free trypsin, centrifuge, and remove the supernatant; the precipitated fraction is the collected cells; resuspend the cells with prechilled 1× PBS solution and centrifuge again to wash the cells; add 300 *μ*L of 1× binding buffer; add 5 *μ*L of Annexin V-FITC for labeling and incubate for 15 min at room temperature, protected from light; add another 5 ul of PI for staining 5 min before loading. Add 200 ul of 1× binding buffer before the machine and detect the apoptosis rate by flow cytometry without light.

### 2.4. Cell Scratching Experiments

After the cells were digested and resuspended, the cells were inoculated in 6-well plates at a number of 6 × 10^5^ cells per well, and the cells continued to be cultured. When the cell confluence was close to 80%, the plate was scratched vertically with a sterilized 100 ul gun tip, followed by washing with PBS three times to remove the scratched cells and then adding serum-free medium to continue the culture. The scratches were observed at 0 h and 24 h, respectively, and photographed. The migration distance was calculated using Nis-Elements BR v.4.30.02 software. The cells were digested with trypsin, resuspended with serum-free medium and counted, and diluted with serum-free medium to ensure that the number of cells in the final 200 ul of cell suspension was 5 × 10^4^. 200 ul of serum-free cell suspension was planted in the upper chamber of transwell cell culture chambers coated with gelatin matrix, and 500 ul of medium containing 20% FBS was added to the lower chamber. After 24 h, the cells in the upper chamber were carefully removed with cotton swabs, and the cells at the bottom of the chamber were fixed with 4% paraformaldehyde and then stained with 0.1% crystal violet for 10 min at room temperature, rinsed, and observed under the microscope and photographed. Before the experiment, the desired well plates and tips were precooled at 4°C, and the matrix gel was dissolved on ice. During the gelation process, the cells were digested and resuspended, and the cell density was adjusted, so that the final number of cells added to each well was 1 × 10^5^. After the cells were added, the well plates were continued to be incubated for 24 h, observed under a light microscope and photographed, and analyzed using Image *J* software. Total cellular proteins were extracted and subjected to protein immunoblotting.

### 2.5. Statistics

All data in the experiment were expressed as mean ± standard deviation (*χ* ± SD), and SPSS 23.0 was used for data processing and analysis. The *t*-test was used for comparison between two groups of samples, and a one-way analysis of variance (one-way-ANOVA) was used for comparison between multiple groups of samples. Significant differences between statistical results were indicated by *P* < 0.05.

## 3. Results

### 3.1. Detection of MMP-10 Interference Efficiency

It transfected the cells with the interfering RNA of MMP-10 and examined the expression of MMP-10 at the protein and RNA levels by Western blot and qRT-PCR, and the results are shown in Figure 1. It could be used for subsequent experiments.

### 3.2. Results of CCK-8 Detection of Cell Proliferation

Figure 2 shows the CCK-8 experimental results. The corresponding OD values were measured at 0 h, 24 h, 48 h, and 72 h of cell culture by coexpressing miR-363 mimic and si-MMP-10, respectively, on top of overexpression of circRNA-0024103, and it was found that overexpression of circRNA-0024103 resulted in a significant enhancement of cell proliferation, while coexpression of miR-363 mimic or MMP-10 siRNA cotransfected with circRNA-0024103 plasmid resulted in abrogation of the proliferative effect induced by overexpression of circRNA-0024103 alone (*P* < 0.05) in human umbilical vein endothelial cells.

### 3.3. EdU Assay Cell Proliferation Results

It was further verified the effect of combining miR-363 mimic and MMP-10, respectively, on cell proliferation ability by EdU assay on top of overexpression of circRNA-0024103. As shown in Figure 4, compared with the control group, the number of EdU-positive cells was significantly increased after circRNA-0024103 overexpression, while the number of EdU-positive cells was significantly reduced after the addition of miR-363 mimic or MMP-10 siRNA, and the proliferation-promoting effect of circRNA-0024103 overexpression was significantly inhibited. The results of the EdU experiment are shown in Figure 3.

### 3.4. Flow Detection of Apoptosis Results

The results of apoptosis detection by flow are shown in Figure 4. The number of apoptotic cells was significantly reduced after cells overexpressed circRNA-0024103, while the number of apoptotic cells was significantly increased after cotransfection of miR-363 mimic or MMP-10 siRNA with circRNA-0024103 plasmid.

### 3.5. Results of Scratch Assay to Detect Cell Migration Ability

We examined the migratory ability of cells by observing the distance and cell number of cell migration and found that after 24 h of scratching, the overexpression of circRNA-0024103 significantly increased the migratory distance and cell number of cells compared with the control group, and the migratory ability of cells was significantly enhanced. The migratory ability of cells was significantly reduced after cotransfection of miR-363 mimic or MMP-10 siRNA with circRNA-0024103 plasmid.

### 3.6. Transwell Assay Results for Cell Invasion Ability

We observed the invasion ability of cells by transwell assay, and the results of cell invasion experiments are shown in Figures 5 and 6. The number of cells invading from the upper chamber to the lower chamber of transwell was significantly increased after overexpression of circRNA-0024103. In contrast, the number of cells invading from the upper chamber to the lower chamber was significantly reduced after the cells were treated with miR-363 mimic or MMP-10 siRNA in combination with overexpression of circRNA-0024103, compared with overexpression of circRNA-0024103 alone.

### 3.7. Results of Cell Tube Formation Experiments

Tube-forming assay is a method to study the ability of cell formation by mixing cells and stromal glue word to simulate the environment of blood vessel formation. As shown in Figure 7, the formation of capillary-like structures was significantly increased after overexpression of circRNA-0024103, and the tube-forming ability of the cells was significantly enhanced, while the formation of capillary-like structures was significantly reduced after treatment of cells with miR-363 mimic or MMP-10 siRNA in combination with overexpression of circRNA-0024103, and the tube-forming ability was significantly weakened.

### 3.8. Effect of circRNA-0024103 Overexpression on VEGF Expression

We examined the effect of circRNA-0024103 overexpression on VEGF expression by Western blot, and the results are shown in Figure 8. circRNA-0024103 overexpression significantly increased the expression of cellular VEGF compared to the control group.

### 3.9. Effect of circRNA-0024103 Silencing on miR-363 and MMP-13 Expression

We silenced circRNA-0024103 by siRNA and tested the effect on the expression of miR-363 and MMP-13.  Figure 9(a) shows that the expression of circRNA-0024103 in cells was significantly reduced after interfering with siRNA, and its interference efficiency was more than 50%. The expression of miR-363 was significantly increased after circRNA-0024103 silencing (Figure 9(b)), while the expression of MMP-10 was significantly decreased (Figure 9(c)). However, the silencing of circRNA-0024103 in combination with the inhibitor of miR-363 reversed the inhibitory effect of circ-0024103 silencing on MMP-10 expression (Figure 9(c)).

### 3.10. Effect of circRNA-0024103 Overexpression on miR-363 and MMP-13 Expression

We achieved overexpression of cellular circRNA-0024103 by transfecting circRNA-0024103 overexpression plasmid and further tested to detect the effect on miR-363 and MMP-13 expression. As shown in Figure 10, the expression of miR-363 was significantly reduced after circRNA-0024103 overexpression (Figure 10(a)), and the expression of MMP-10 was significantly increased (Figure 10(b)), while the simultaneous intervention with mIR-163 mimic reversed the increase of MMP-10 caused by circRNA-0024103 overexpression (Figure 10(b)).

### 3.11. CircRNA-0024103 Regulates VEGF Expression in HUVECs after ox-LDL Induction via miR-363/MMP-10 Axis

We combined different interventions based on overexpression of circRNA-0024103 to observe the effect on cellular VEGF expression. The results showed that overexpression of circRNA-0024103 increased VEGF expression, while combining miR-363 mimic or MMP-10 siRNA reversed the increase in VEGF caused by circRNA-0024103 overexpression (Figure 11).

### 3.12. Results of Luciferase Reporter Gene Experiments

To further reveal the regulatory relationship of circRNA-0024103 on miR-363, we inserted the full sequence of circRNA-0024103 into the luciferase reporter and found that the luciferase activity of the wild-type (circRNA-CRE WT) was significantly reduced after miR-363 mimic treatment. However, no significant change was found in the activity of the mutant (circRNA-CRE Mut) compared with the control (Figure 12(a)), suggesting a direct binding between the two. Similarly, we tested whether miR-363 interacted with the target gene MMP-10 by the same method and found that the luciferase activity was significantly decreased in the wild-type (MMP-10 WT), and no significant change was found in the mutant (MMP-10 Mut) luciferase activity (Figure 12(b)), suggesting a direct binding between the two.

## 4. Discussion and Conclusion

CircRNA exerts its biological functions in many ways, among which the most studied is its role as a miRNA sponge. circRNA can act as a competitive binding miRNA for 0024103NA and as a miRNA sponge to silence miRNA, so it can act as a regulator of transcription or translation, affecting the splicing of precursor mRNAs, and then participate in protein translation and other processes, playing regulatory roles in different stages of organism development and pathophysiological processes. For example, circRNA (HRCR) can act as a sponge for miR-223, thereby inhibiting miR-223 activity and exerting its protective role in cardiovascular diseases [4]. hsa_circ_0007623, as a sponge for miR-297, can promote cardiac repair after acute myocardial ischemia by upregulating vascular endothelial growth factor-A expression.

In the previous section, we demonstrated that circRNA-0024103 regulates VEGF expression in endothelial cells via miR-363/MMP-10 axis, and circRNA-0024103 can function as a sponge for miRNA-363 and MMP-10. Therefore, in this part of the experiment, we further observed the effect of circRNA-0024103 modulating the miR-363/MMP-10 axis on the biological behavior of endothelial cells such as proliferation and migration after ox-LDL induction. We examined the proliferative capacity of cells by CCK-8 and EdU assays and showed that miR-363 mimic or MMP-10 siRNA significantly attenuated the proliferation-promoting effect of overexpression of circRNA-0024103 on cell proliferation. In the flow cytometry assay of apoptosis, overexpression of circRNA-0024103 inhibited the apoptosis of endothelial cells, and the intervention of combined miR-363 mimic or MMP-10 siRNA counteracted the inhibition of apoptosis by overexpression of circRNA-0024103, resulting in a significant increase in the number of endothelial cells undergoing apoptosis [13]. Furthermore, we explored the effects of circRNA-0024103/miR-363/MMP-10 regulatory axis on endothelial cell migration, invasion, and tube-forming ability by cell scoring assay, transwell assay, and tube-forming assay, respectively. The migration, invasion, and tube-forming ability of endothelial cells were significantly enhanced by overexpression of circRNA-0024103, while the promotion effect of overexpression of circRNA-0024103 alone on migration, invasion, and tube-forming ability was counteracted when combined with miR-363 mimic or MMP-10 siRNA.

In conclusion, our results suggest that circRNA-0024103 exerts regulatory effects on the biological behaviors of endothelial cells, such as proliferation, apoptosis, migration, and invasion, by regulating the miR-363/MMP-10 axis. This contributes to the refinement of the role of circRNA in atherosclerosis. The results of this part of the experiment showed that circRNA-0024103 regulates biological behaviors such as proliferation, apoptosis, migration, and invasion of endothelial cells through the miR-363/MMP-10 axis. However, our findings cannot specifically illustrate the functional mechanism of circRNA-0024103 in atherosclerosis. We still need to do more experiments in the future.

## Figures and Tables

**Figure 1:** Western blot and qRT-PC detection of MMP-10 expression after interference.

**Figure 2:** CCK-8 experimental results (^*∗*^*P* < 0.05 vs. the control group).

**Figure 3:** Results of the EdU experiment (^*∗*^*P* < 0.05 vs. control).

**Figure 4:** Results of apoptosis detection by flow (^*∗*^*P* < 0.05 vs. control).

**Figure 5:** Results of scratch experiments (^*∗*^*P* < 0.05 vs. the control group).

**Figure 6:** Results of cell invasion experiments (^*∗*^*P* < 0.05 vs. control).

**Figure 7:** Results of the tube formation experiment (^*∗*^*P* < 0.05 vs. the control group).

**Figure 8:** Effect of circRNA-0024103 overexpression on VEGF expression.

**Figure 9:** Effect of circRNA-0024103 silencing on miR-363 and MMP-13 expression (^*∗*^*P* < 0.05 vs. the si-NC group).

**Figure 10:** Effect of circRNA-0024103 overexpression on miR-363 and MMP-13 expression (^*∗*^*P* < 0.05 vs. control).

**Figure 11:** CircRNA-0024103 regulates VEGF expression through the miR-363/MMP-10 axis.

**Figure 12:** Results of luciferase reporter gene experiments.

**Table 1:** Primer sequences.

Name (of a thing)	Primer sequences (5′ to 3′)
circRNA-0024103	Forward: CTGGTGCAGTGGAAGCAGAG
	Reverse: CGACCCTCCATTGCTCTTCT

U6	Forward: TGCGGGTGCTCGCTTCGCAGC
	Reverse: CCAGTGCAGGGTCCGAGGT

## Data Availability

The datasets used and/or analyzed during the current study are available from the corresponding author upon request.
